# Construction and Application of a Piano Playing Pitch Recognition Model Based on Neural Network

**DOI:** 10.1155/2022/8431982

**Published:** 2022-09-17

**Authors:** Guobin Wu, Wei Chen

**Affiliations:** Changchun Humanities and Sciences College, Changchun, Jilin 130117, China

## Abstract

The intonation recognition of piano scores is an important problem in the field of music information retrieval. Based on the neural network theory, this study constructs a piano playing intonation recognition model and uses the optimized result as the feature of piano music to realize the prediction of the music recognition of the intonation preference. The model combines the behavioral preference relationship between intonation and musical notation to measure the similarity between intonations, which is used to calculate the similarity between intonation preference and music, and solves the quantification problem of intonation recognition. In the simulation process, the pitch preference feature of piano playing is used as the identification basis, and the effectiveness of the algorithm is verified through four sets of experiments. The experimental results show that the average symbol error rate of the improved network model is reduced to 0.3234%, and the model training time is about 33.3% of the traditional convolutional recurrent neural network, which is optimized in terms of recognition accuracy and training time in single-class pitch feature. In the recommended method of multi-category evaluation of pitch features, the recognition accuracy of multi-category pitch features is 42.89%, which effectively improves the musical tone recognition rate.

## 1. Introduction

With the rapid growth of the number of digital music, the piano playing pitch recognition algorithm performs personalized identification by analyzing the historical behavior of pitch-on-demand music [1]. As a hotspot of development in the new century, the neural network has gained more and more attention and application depending on its advantages in nonlinearity, self-learning, robustness, and self-adaptation [2–4]. As one of the most successful models of neural networks, the BP network has been able to simulate complex nonlinear models by virtue of its powerful nonlinear mapping capability, parallel distributed processing capability, adaptive capability, fault tolerance capability, and generalization capability [5]. The error is minimized; therefore, we adopt the BP network as the reference model for musical tone recognition [6].

Traditional machine learning techniques are limited in processing natural data in its raw form [7]. For a long time, the construction of recognition models is very difficult and requires considerable time and effort to complete [8]. In addition, professional knowledge in related fields is also essential, because feature extraction classifier needs assistance [9–11] to perform effective analysis and appropriate feature representation on the original data (such as image pixels and audio signals) [12] for the classification subsystem to analyze the input raw data, and the complexity of the original data requires a lot of time and effort to analyze, and the analysis results are difficult to apply to other data scenarios [13].

In this study, a piano playing intonation recognition model is constructed, and the tool is used to generate the spectrum of piano music. Four music categories are set: blues, classical, jazz, and pop. For the training of CNN (convolutional neural network), two activation functions, ELU (exponential linear unit) and ReLU (rectified linear unit), and two gradient descent methods were explored. Experiments show that ELU is more stable than ReLU, and Adam has faster gradient descent than RMSProp. Comparing the classification methods based on the spectrum, the latter has an improvement of 1.5% on the basis of the former's classification accuracy of 96%. In addition, aiming at the problem of octave interference in the existing autocorrelation identification method, an improved note identification method is designed using the frameshift method. Taking the comprehensive features as the classification basis, the automatic recognition method of notes is explored as an explicit classification feature.

## 2. Related Work

The piano tone signal is composed of the fundamental tone and the overtone [14]. Due to the significant differences between Western music and Chinese music in musical styles and modal systems, each has its own independent system in music theory: therefore, the modal tonality analysis module also treats Western music and folk music separately. The output of the module is a clear textual representation indicating the modal key of the music entered into the module for analysis [15].

Román et al. [16] proposed a research method on music score images, including digitization, recognition, and restoration, and summarized the software and hardware required by the pitch recognition system, explored potential application scenarios of pitch recognition, and promoted pitch recognition identification research. Nakamura et al. [17] used a neural network model for optical score recognition and gradually adopted an end-to-end piano score recognition method to simplify the research method based on a general framework. Segmentation is achieved using the region growing method and improved Hough transform detection for the fringes, and the rest of the notes are extracted again through template matching. Watts [18] used a multi-track data set to train and test the model, using a convolution-recurrent neural network that effectively learned both spectral features and audio contextual information. The creative achievement of Qian et al. [19] is mainly to achieve as many as 18 instrument categories at the same time, which also includes the identification of male singers (tenor and bass) and female singers (soprano and alto). The recognition of pure musical instruments also achieves high accuracy.

Although the staff information is the auxiliary information of the note, that is, the position of the note in the staff determines its pitch and other information, to a certain extent, the existence of the staff will interfere with the identification of the note, so the accuracy of staff detection and deletion will directly affect the note [20]. However, the cross-overlapping characteristics of staff and notes make it difficult to delete staff. When the staves are not deleted enough, the remaining staves will affect the recognition of notes. Combining collaborative filtering with intonation context information, the original intonation data scoring model of collaborative filtering is extended to form a three-dimensional data model of intonation-data-context, which expands the correlation dimension and achieves more accurate personalized recognition [21]. In this indirect identification scheme, although there is no correlation between users and data, a third party can be used [22]. Because of the strong correlation between notes, the reconstruction of notes needs to incorporate contextual information. It is not only necessary to combine the relevant information of the staff but also inseparable from the time signature, key signature, clef, and other information in the music score, and grammar-based reconstruction can effectively solve this problem.

## 3. Construction of a Neural Network-Based Piano Playing Pitch Recognition Model

### 3.1. Hierarchical Distribution of Neural Network

The neural network only needs to build a suitable learning network, and multiple hidden layers in the network will automatically learn various features, and there is a progressive relationship between the hidden layers, and the latter layer is a more abstract description of the previous layer. The neural network generally consists of three parts: first, the input layer *x* (*c*, *s*); second, the hidden layer *v* (*x*); the neural network obtains the features of each part of the original data samples and further compresses and abstracts the features. Third, the output layer *g* (*x*−*x*') compares and classifies the feature results, compares the expected results during training, back propagates the error of the results, and calculates the probability *y*−*s* of each classification during prediction.

(1) $$\begin{array}{c} \frac{1-x\left(c,s\right)}{N}=\sum \ln\;\left(c-1\right)-r\left(y-s\right)\text{,}\\ \partial \beta \left(x\right)v\left(x\right)-y\left(1-\beta \right)\left(g\left(x-x^{\prime }\right)\right)-1=0\text{.} \end{array}$$

Each node of the hidden layer represents a neuron, each arrow represents a feature transfer function *r* (*c*, *s*) of the data, and the weight carried by each function represents the neuron's “perception” of the data *k*, and finally, the weight sim (*c*−1) is adjusted by the error fed back by the output layer, making the neuron's “perception” of the data more accurate. To control each training error sim (*c*−*s*), the gradient descent method is generally used to ensure that each iteration training can reduce the error.

(2) $$\begin{array}{c} \bar{r\left(c,s\right)}-r\left(c,s\right)=\left\{\begin{array}{c} k\sum sim\left(c-1\right)\\ 1-sim\left(c-s\right) \end{array}\right.\text{,}\\ \frac{1}{2}k=\frac{1}{\sum sim\left(x\right)}-di\;am\left(x\right)-\left|sim\left(x\right)\right|\text{.} \end{array}$$

However, activation functions sim (*x*) such as rectified linear units that introduce sparsity by reducing the coupling ability in certain ranges are equivalent to pre-training in unsupervised learning diam (*x*). The starting point of the horizontal line on the lower side of the center line of the long ruler was located to the left of the starting point of the horizontal line on the upper side of the center line of the time length ruler, indicating that the note was sung fast.

Obviously, the amount of data after the pooling operation s (*x*) *c* (*x*) is reduced to a quarter of the original. The feature map *c* (*x*) obtained after the pooling operation is reduced in dimension compared with the original, which realizes the network dimension reduction.

(3) $$\begin{array}{c} y=\left\{\begin{array}{c} \sum c\left(x\right)-\left|c\left(x\right)\right|\text{,}\\ 1-\left|s\left(x\right)c\left(x\right)\right|\text{,} \end{array}\right.\\ C=1-\left|c\left(1\right),c\left(2\right),c\left(3\right),c\left(4\right),\ldots ,c\left(x\right)\right|\text{.} \end{array}$$

Since the statistical characteristics of one part of the image are the same as other parts, the features learned from one part can also be used in another part, so a convolution kernel can share the same set of parameters in the process of convolution of the input lim (*x*). To further compare the features, a pooling operation sim (*x* (*i*)) is performed after the convolution. That is, the actual output of each output unit in the neural network is basically consistent with the expected output.

(4) $$\begin{array}{c} \lim_{x⟶\infty }\left[\frac{1}{n}\sum sim\left(x\right)-sim\left(x-1\right)\right]-\sqrt{sim\left(x\left(i\right)-x\right)}=0\text{,}\\ F\left(x,a\right)\in f\left(a,n\right)-2^{1-n\;\sin\;\theta }\text{.} \end{array}$$

The purpose of learning and training the neural network *F* (*x*, *a*) is to construct the inner connection *f* (*a*, *n*) and law of the musical sound signal through the training sample library, that is, to construct the basic model of recognition. The output layer number of nodes is the same as the number of hidden layer nodes, that is, the number of categories of piano monophony. For the identification of musical tones, we can divide it into t-ends and use the corresponding model.  Figure 1 achieves the purpose of music segmentation optimization by calculating its small cumulative prediction residual.

The objects analyzed by the mode key analysis module cover most of the music—Western tonal music and national modes. The input of the module is the output (result) of the feature extraction module of the pitch and duration of the monomelody music, and of course, it can also be a two-dimensional array containing pitch and duration information. The difference in harmonic structure is mainly reflected in the first three-order harmonics, and the energy distribution of the latter harmonics with higher orders is similar, so when paying attention to the first three-order harmonics, the identification score is the highest, and the number of harmonics concerned is the highest.

### 3.2. Frequency Domain Classification of Piano Playing

First, we need to construct a baseline model for musical instrument recognition as a basis for subsequent model improvements and experimental comparisons. We adapt the proposed neural network model, which has been shown in the literature to be effective for the problem of automatic music labeling. Furthermore, we use training data with frame-level precision labels as supervision signals for training the network, while they train the model in a weakly supervised manner. The ratio *s* (*i*) of the sampling frequency to the pitch period is the pitch frequency, and there is a one-to-one correspondence between the pitch frequency and the note.

(5) $$\begin{array}{c} S\left(i,j\right)=\left\{\begin{array}{c} s\left(i\right)|i=1,2,3\ldots ,n\text{;}\\ s\left(j\right)|j=1,2,3\ldots ,n\text{,} \end{array}\right.\\ \frac{1}{3}\left(h\left(\theta ,x\right)-h\left(x\right)/i>0\right)-\bar{h\left(x,y\right)-y{\left(i\right)}^{2}}=1\text{.} \end{array}$$

It can be seen that if you want to obtain the frequency value *h* (*x*)/*i* of a certain time period *i*, you need to count the number of all frequency values in this time period and select the largest number as the frequency value of this time period *h* (*x*, *y*). The shorter the time period, the more accurate the frequency value of the time period. Doing this every other time period, sim (*r*) produces a graph of the frequency distribution *c* (*i*, *j*) over time. If the amplitude feature *a* (*x*) is added to the spectrum, a multidimensional spectrum can be obtained.

(6) $$\begin{array}{c} \left\{\begin{array}{c} 0<sim\left(r,c\left(i-1,j-1\right)\right),\\ 0<\sum sim\left(r,c\left(i,j\right)\right)*r\left(c-s\right), \end{array}\right.\\ \theta \left(i,x\right)-a\left(x\right)\frac{\partial a/i}{\partial i}-\bar{i\left(x,y\right)-j\left(i\right)}=1\text{.} \end{array}$$

Note pitch frequencies are compressed vertically to 128 levels, and grayscale levels are also 256 levels, where *p* (*r*) is the expectation factor. The first condition for the above formula to be established in the system is that the process is stable. For the specific training method, we can choose the optimal gradient descent method. The instantaneous value of *b* (*g*−*r*) at the time gate is used to replace the sum *x* (*r*−*b*) of squares of errors to solve the defects of the statistical characteristics of the objective function *a* + *r* of the whole system at one time.

(7) $$\begin{array}{c} \left\{\begin{array}{c} y\left(p\left(r\right)+1-b\left(g-r\right)\right)\geq g,\\ x\left(r-b\right)\geq g, \end{array}\right.\\ \Delta \theta =1-\frac{\alpha -r}{\partial a+r}-x\left(r-b\right)-g\text{.} \end{array}$$

Because of its segmented and derivable advantages, it is applied to practical problems. The nonlinear characteristics enhance the fitting ability *x* (*r*−*b*) of the function to the data, and the linear characteristics in the range of positive real numbers make the gradient calculation of the model simple and fast during the training process.

The input layer and the hidden layer are fully connected, but the weight is fixed at 1. There is no need to pre-determine the weight between the hidden layer and the output layer, and it can be calculated directly in the next step. According to the scheme, in order to facilitate setting the threshold value and enhance the signal's adaptability to the signal, we first normalize the signal, then divide the data into frames, and obtain its short-term energy and short-term zero-crossing rate frame by frame, and we set two threshold thresholds.

Figure 2 “forces” the convolution by constructing a harmonic sequence matrix to focus on the corresponding number of harmonics in the process of learning intermediate features. The nodes are discarded directly, and only the parameters between the solid line nodes are learned; that is, the state transition matrix of this model is sparse, which reduces the computational complexity of model training. In each round of training, nodes are randomly selected in a certain proportion, and the remaining node information is discarded. Since the nodes removed in each round are not fixed, it is equivalent to training different models with the same data, and the results will be more accurate when integrated, which effectively alleviates the huge amount of parameter calculation introduced by the full connection. However, due to the complexity of the performance situation, the situation of playing wrong is also intricate, for example: playing a few bars of notes, and the subsequent bars are all correct; this situation will be considered by the system: starting from the first bar where the error occurs.

### 3.3. Pitch Recognition Feature Extraction

In the process of recognizing multiple pieces of piano music, it was found that when the rhythm of the piano music was slow, that is, when the number of notes per second was less than 2, the recognition accuracy of both was very high; when the number of notes per second was in the range of 2∼4, the recognition accuracy rate of the traditional method begins to decline, but the improved algorithm can still ensure high accuracy; when the number of notes per second exceeds 5, it means that the interval between each two notes is less than 0.2 seconds, which will lead to harmonics of the previous note. The wave has not decayed enough to interfere with the harmonics of the latter note, so neither method has a high rate of recognition. Under normal circumstances, the number of notes per second in piano music is in the range of 2 to 3, and the number of notes per second over 5 usually only occupies a small section, so the improved algorithm can basically meet the classification requirements.

This model is developed on the basis of the left-to-right model without spanning, which allows the state to jump at intervals, and describes the phenomenon that some pronunciation units in speech are absorbed or deleted in actual speech. For a more complex model, there are two parallel branches, and jumps are also allowed between the branches. Based on the aforementioned research, we choose an extraction algorithm with better performance, MFCC (Meier cepstral coefficient) feature extraction algorithm to process the signal. The specific extraction results are shown in Figure 3.

Through analysis, we select LPCC (linear prediction cepstrum coefficient) and feature parameters extracted by the MFCC algorithm as the input vector of BP network. After that, we normalize the input data, so that some abnormal input can fall within the expected range, and strengthen the adaptability of the system to musical sound data.

According to the different calculation methods of intonation preference features, this study proposes a recognition method for comprehensive evaluation of user features and a multi-category evaluation method for intonation features and makes an experimental comparison between the two methods. The experimental results show that the recognition method of comprehensive evaluation of intonation features is suitable for the recognition of single-class intonation, while the recognition method of multi-class evaluation of intonation features is suitable for the recognition of multi-class intonation. On the whole, the recognition result of comprehensive evaluation of intonation features is better than that of intonation.

### 3.4. Neural Network Data Convolution

The signal was acquired and saved with the file name “elise. wav.” Then, we use the program to read it into MATLAB. In the abovementioned recognition system using the 88 key tones of the piano as the sample training library, we constructed the signal recognition model through signal preprocessing and feature extraction. On the basis of again, we conducted a comparative experiment on the extraction methods of hidden layer neurons and feature parameters and selected the optimal number of hidden layer neurons and a feature parameter extraction scheme with better performance.

One of the most useful properties of this feature vector is as follows: it can encode the chords contained in a given song. Therefore, two audio frames with similar harmonic content will have the same feature vector. There is a positive correlation between the pitch estimation effect and the instrument recognition effect. It can be seen that after the completion of 200 epochs of AlexNet and its improved network, the spectral recognition accuracy of the verification set music tends to be stable, and the verification set spectral recognition accuracy of AlexNet-improved-v2 has reached the highest. The spectral recognition accuracy of the validation set is 1.08% higher than that of AlexNet-improved-v1 and 1.90% higher than that of AlexNet. Based on the experiments in Figure 4, AlexNet-improved-v2 is more suitable for the music genre recognition model.

Like single-note recognition preprocessing, continuous tones also need to undergo signal de-noising, endpoint detection, and single-note segmentation, but the difference from the single note is that the endpoint detection and signal segmentation of the single note are mainly to further simplify the signal, increase the proportion of useful information, and improve the recognition accuracy of the system; the recognition of continuous musical tones is to extract the continuous signal from the continuous signal. In addition, since timbre and dynamics are relative quantities, it is not convenient to compare, only the corresponding information is extracted, and this factor is not considered in the comparison and results. This function can be improved in future research and expansion. With this feature vector, we can calculate the correlation of the feature vectors of the two audio frames and measure the similarity of the two audio frames accordingly.

### 3.5. Similarity Error Analysis

The experimental environment is the same as that of the pitch feature extraction experiment. We divided the Bach10 data set, the Mixing Secrets data set, the MedleyDB data set, and the self-built data set, four data sets with annotation labels of frame-level instrument activity levels, into training and test sets in a ratio of 9 : 1, respectively. The audio data for the four categories were segmented to obtain approximately 8000 fragment image samples each. 40% of the image samples are used as training samples, 30% are used as verification samples, and 30% are used as test samples.

For the network optimization of the first-level classification model, Figure 5 uses the algorithm with a momentum of 0.9, a mini-batch size of 100, an initial learning rate of 0.05, and a weight decay factor of 4. For each residual network in the second-level classification model, the network was optimized using the algorithm with a momentum of 0.9, a mini-batch size of 64, and an initial learning rate of 0.1, and it divides the learning rate by 10 every 30 epochs and set the max training epochs to 100 and weight decay to 4. The scene text classification module uses the convolutional neural network technology to identify the business scene of the input text sequence, and the named entity recognition module receives the scene and text sequence from the scene text classification module and uses the NER model based on the composite framework to identify the named entity.

For the needs and convenience of research, many scholars do not consider diminished chords. For each scale, this article defines major chords, minor chords, diminished chords, and three categories of 36 chords according to their names. Experiments found that this set of chord types is appropriate, and it is between over-learning and under-learning. This shows that when the number of windows is the same, the entropy sequence output of the spectrum obtained is basically the same, but when the difference in the number of windows is large, the obtained entropy sequences are slightly different. After experimental verification, when the difference in the number of windows is greater than 30, the obtained entropy sequence has a large difference. Thus, it was concluded that when the number reached 20, the number of neurons increased, although it takes more system training time, the recognition performance cannot be improved again.

## 4. Application and Analysis of Piano Playing Pitch Recognition Model Based on Neural Network

### 4.1. Neural Network Data Preprocessing

100 experimental samples were tested, 82 samples with recognition rate above 9 s%, 1 sample with recognition rate lower than 50%, and 6 samples with recognition rate lower than 70%. Observing the samples in which the R chord is less than 70% of the experimental results, it is found that such experimental samples belong to absolute consonant chords in music, and the two-tone interval is more than 13° apart: that is to say, this module has absolute consonant interval resolution for polyphonic intervals. The presentation layer is mainly the interface for the direct interaction between users and the system. The user can input text sequences through this module and then perform operations on viewing named entities; the logic layer is the business processing part of the entire system, which implements all the logical functions of the system, mainly including scene text.

It can be seen that the musical tone recognition system of Figure 6 has a high musical tone recognition efficiency, which basically meets the requirements for the main frequency of musical tones. However, we also see that due to the longer length of the last note of the elise continuous tone, the proportion of its overtone in the tone signal increases, which has a certain impact on the identification of the fundamental tone, and a certain error occurs in the system. When the minimum Euclidean distance is greater than 0.45, most of the speech entropy sequences in the template library with the smallest Euclidean distance from the test template entropy sequence as the recognition result are wrong. Therefore, in this experimental system, the threshold for judging the recognition result is set to 0.45. When the minimum Euclidean distance is greater than 0.45, the recognition result cannot be obtained; when the minimum Euclidean distance is less than 0.45, the speech signal represented by the entropy sequence of the minimum Euclidean distance in the template library is returned. From the prediction results, the system fully meets the identification accuracy requirements. After we get the main frequency of the musical note, we can complete the simple score identification of musical notes through the one-to-one correspondence between the musical note name and the main frequency.

### 4.2. Simulation of Piano Playing Intonation Recognition

The experimental environment of this study is as follows: Ubuntu 16.04 operating system, Intel Core i7-8700 CPU, 16G running memory, Nvidia GTX 1080Ti GPU, and TensorFlow deep learning framework. The model is optimized by the Adam adaptive learning rate algorithm during the training process, which combines the momentum-based algorithm and the adaptive-based algorithm and sets the initial learning rate to 1e-3 and the batch size to 16. In the next iteration, the algorithm evaluates the symbol error rate on the validation set to verify the accuracy of the model.

The system distinguishes and recognizes chords by distinguishing different states. A model is a stochastic finite state machine in which each state produces an observation. The music crawler system can download music on the Internet in batches to build a self-built data set based on the Internet music library to improve the robustness of the music genre identification system.

The network output in Table 1 is converted to the conditional probability distribution on the label sequence. The two-tone pitch duration extraction module accurately reflects the chord duration and pitch information. Since the analysis window is deterministic, if the input is a fast-paced segment, it means that the window will span more notes, and a frame of data is likely to contain more than one type of chord, thus confusing the system. Through this module, the pitch and vibration time of two-tone chords can be analyzed. Through the work of this study, the work of comparing musical scores and audio files has been transformed into a relatively mature string search and comparison work with the help of music feature extraction. It can be expected that if algorithms such as fuzzy search are used for this matching and comparison. More precise conclusions will be made for more performance situations.

First, the C-BiLSTM is trained in the data set in Figure 7, and its effectiveness is verified by comparing the recognition error rates before and after image enhancement; then, the CNN is improved to a residual CNN and its effect on the generalization ability of the model is verified. Secondly, a multi-scale fusion algorithm is added to the residual CNN, and its influence on the feature extraction ability of the model is proved by comparing the feature maps of each convolutional layer of the model and the symbol error rate.

The half-part structure is the top-down feature fusion part, and the pixel-level fusion of the deeper feature map C5 containing semantic information and the upper-level feature map C4 is performed, because the fusion requires the two feature maps to maintain the size and dimension, so the size of C5 is kept consistent with the size of the feature map C4 through 2 times upsampling, and the feature map C4 is passed through a 1 × 1 convolution kernel to ensure that the feature dimension after upsampling is the same as that of C5, and the feature map F5 is obtained after fusion. The same is done for feature maps F5 and C3, and finally, feature map F4 is obtained. As a result, features containing different levels of information are obtained, to achieve multi-scale feature fusion, so that the feature vector used in subsequent note recognition contains more detailed and comprehensive information.

### 4.3. Example Application and Analysis

The CNN in the C-BiLSTM network is improved to a residual CNN to form a residual convolutional cyclic neural network, namely RC-BiLSTM. In the same experimental environment, the performance of the model before and after the improved CNN was compared, and the C-BiLSTM network and RC-BiLSTM were trained separately and their symbol error rates were compared. The change in the loss function value of the two networks with the number of iterations during the model training process is shown in the figure, which shows that the loss value of each iteration of the RC-BiLSTM network is lower than that of the C-BiLSTM network, and the loss value of the RC-BiLSTM network has been reduced to 5 and stabilized, while the C-BiLSTM network has only dropped to around 10 with large fluctuations all the time. A collection of neurons is called a layer. On this basis, the outermost layer used for input in the network structure is called the input layer, and the layer used for the final output is called the output layer.

First, we perform feature parameter calculation based on the LPCC (linear prediction cepstral coefficient) algorithm. Using the specific execution steps of the introduced algorithm, considering the accuracy of musical tone recognition and the unity of opposites between the amount of calculation, we choose to use the 12th-order LPCC extraction algorithm, the audio signal FFT (fast Fourier transform algorithm) transformation length is set to 256, the sampling frequency is 20500 Hz, and the length of each frame is 256 points. Through initialization and determination of algorithm prediction coefficients, the feature parameter extraction based on the LPCC algorithm is completed, and 6-frame feature parameters are taken in Table 2.

At the same time, the symbol error rates in the two algorithms are compared in the validation set after every 1000 iterations, and the results are shown in the following figure. During the entire training process, the symbol error rate of the C-BiLSTM network dropped to a minimum of about 4%, but at about 5.2 × 10^4^ iterations, the symbol error rate increased significantly, showing that the model did not converge, while the symbol error rate of the network can be stably reduced to less than 2%, and the fluctuation is small. It can be seen that the accuracy of RC-BiLSTM network note recognition has been significantly improved.

This shows that residual CNN can not only improve the accuracy of the model but also solve the problem of model degradation and enhance the generalization ability of the model. For the MFCC feature parameter extraction method, to facilitate the comparative analysis, our parameter settings are the same as the LPCC algorithm and then the DCT (discrete cosine transformation) parameter solution, pre-emphasis filter filtering, and musical sound signal are go troughed. The frames are further divided, and finally, the MFCC parameters of the musical sound signal are calculated. The data set provides the original quartet chorus pieces, and we can generate more recordings with a different polyphony by exploring the different combinations of voices in each piece. The performance dynamics of these new recordings are the same as the original recordings, providing instrument recognition algorithms with samples of multi-instrumental performance test data at a different polyphony.

The comparison of the recognition results of the two recognition methods for different pitch types is shown in Figure 8. The string matching method is to use strings to represent the melody and then uses string retrieval, quick matching, and other methods to match, by retrieving from the database the characteristic strings of the humming melody. It can be seen that the experimental results and the theoretical values have a good approximation. The experimental data are still derived from the performance of piano players. However, the data used in the module test are the basic two-tone chords in music, and they will not change after the vibration is triggered; that is, they are stable on two tones. To test the performance of this module, 100 two-tone chords with different ranges, different spans, and different degrees of consonance were selected. If the time value feature is further normalized and the length of the sound is specified with a strict musical time value concept, it can be obtained. Here, the normalization method is to take the duration of each note played as the smallest duration unit (such as a quarter beat) as a metric and take its proportional value. Compared with capella-scan, the recognition effect of tuplets and ties is poor. When the algorithm in this study is large, there will be serious errors in simple note recognition, and when the note occupies more pixels, the recognition rate is significantly improved.

## 5. Conclusion

Based on the neural network, this study constructs a piano playing intonation recognition model and uses the optimized classification result as the classification feature of piano music. The interaction between the user and the system includes two use cases of inputting text sequences and viewing named entities. The viewing named entity use cases include scene text classification and named entity recognition. These four use cases provide their own functions for obtaining named entities of text sequences, so that users can accurately obtain the required data information. First, image enhancement is performed on some score examples in the data set to expand the score image data and improve the robustness of the training model. By analyzing the LPCC feature parameters and MFCC feature parameters, through the analysis and comparison of their principles, the superiority of the MFCC feature parameters in musical tone recognition is determined. Named entity recognition receives business scenarios from scene text classification and selects the corresponding NER model. The NER model is trained based on the composite framework of transformer network and recurrent neural network. The NER model is used to identify named entities in text sequences and feedback to users. Using the heuristic estimation algorithm when estimating pitch offset, this dynamic programming-based method can meet the requirements of people with general humming level, but the dynamic programming method takes a long time to match large amount of calculation. The results show that the accuracy of the recognition method in this study is more than 50%, which is close to the performance level of similar international methods. The identification method in this study still has a certain gap and needs to be improved.

## Figures and Tables

**Figure 1:** Distribution of cumulative residuals of neural network hierarchical signals.

**Figure 2:** Frequency domain structure of piano playing.

**Figure 3:** Pitch recognition feature extraction distribution.

**Figure 4:** Accuracy of neural network data recognition.

**Figure 5:** Analysis of intonation similarity error of piano playing.

**Figure 6:** Music tone recognition efficiency of neural network data.

**Figure 7:** Pitch recognition topology based on neural network.

**Figure 8:** Framing of the intonation characteristic parameters of piano playing.

**Table 1:** Piano pitch recognition algorithm.

Piano pitch network output	Recognition algorithm codes
Pbestmax = popmax;	Obtain the final target
Pbestmin = popmin;	In the next iteration *p*(*r*)
[newpopmax, newvmax] = updatepop (popmax, vmax);	To verify Δ*θ*
[newpopmin, newvmin] = updatepop (popmin, vmin);	The accuracy *sim*(*x* − 1)
V [*v* < rangespeed [0]] = rangespeed [0]	On the validation set
V [*v* > rangespeed [1]] = rangespeed [1]	Most likely label *x*+*y*
For *j* = 1: popsize	The algorithm evaluates *g*(*x* − *x*′)
If newvalue_max (*j*) > value_max (*j*)	Case of the model
Pbestmax(:, j) = newpopmax (:, j);	By selecting the *α* − *r*
Gbestvaluemax = newgbestvaluemax;	The symbol error rate
Gbestmax = newgbestmax;	*b*(*g* − *r*)
End	For the given input sequence

**Table 2:** Calculation of musical notation characteristic parameters.

Musical notation index	Feature number	Feature percentage	Root mean square	Error rate
Parameter 1	42	86.46	0.52	0.03
Parameter 2	83	42.91	0.07	0.01
Parameter 3	57	48.95	0.29	0.01
Parameter 4	56	96.70	0.06	0.07
Parameter 5	99	62.58	0.35	0.02
Parameter 6	66	65.67	0.24	0.01

## Data Availability

The data used to support the findings of this study can be obtained from the corresponding author upon request.
